# A Diagnostic Model of Volleyball Techniques and Tactics Based on Wireless Communication Network

This article has been retracted.

**DOI:** 10.1155/2022/2185908

**Published:** 2022-03-30

**Authors:** Zhigang Yuan, Yongkui Zhang, Bo Li, Xinlong Jin

**Affiliations:** ^1^Volleyball Teaching and Research Office, Harbin Sport University, Harbin, 150000 Heilongjiang, China; ^2^China Volleyball College, Tianjin University of Sport, Tianjin 300000, China; ^3^Academic Affairs Office, Dalian University of Science and Technology, Dalian, 116000 Liaoning, China

## Abstract

Volleyball is a sport of teamwork competition and tactical coordination. It tests the ability of team members to cooperate with each other and personal resilience. With the development of wireless communication networks, how to use wireless communication networks in the analysis of volleyball tactics is the subject of this article. To explore how to design the volleyball tactics analysis model of the wireless communication network, this paper proposes the method of LTE system and MIMO technology and designs the tactics analysis model based on the characteristics of the wireless network, then combined volleyball tactics and game theory to design a wireless communication network volleyball tactics analysis model. Then, this paper designs the simulation experiment of scene allocation problem, the algorithm simulation experiment, and the comparative investigation and analysis of volleyball game spiking technical ability. The results of the experiment are optimized for the tactical analysis model, and finally, the improvement of the training of the volleyball tactical analysis model based on the wireless communication network is verified through comparative experiments. The experimental results show that the team fit of the volleyball tactical analysis model training based on the wireless communication network has increased by 22.12% compared with the traditional volleyball tactical training. Compared with the traditional volleyball tactical training, the personal on-the-spot adaptability of the volleyball tactical analysis model training based on the wireless communication network has increased by 9.05%.

## 1. Introduction

In recent years, the domestic communication industry has developed rapidly, and earth-shaking changes have occurred in both the technical field and the market field. The importance of wireless communication network planning has increased day by day. With the establishment of the L company, the old wireless communication network planning methods can no longer fully meet the requirements of the times. Discussing how to apply the wireless communication network to the analysis of volleyball tactics, to greatly improve the flexibility and technicality of volleyball tactics, will have important theoretical and practical significance.

This article will rank the technical index data of attack and defense, analyze the ranking of related teams, and have a more accurate and detailed understanding of the technical factors affecting volleyball competition. The participating teams are divided into groups, the attack and defense skills are compared and analyzed, the advantages and disadvantages of traditional volleyball tactics are found, and the disadvantages of traditional volleyball tactics duel in the game are analyzed. The volleyball tactics analysis model designed through the wireless communication network can effectively improve the volleyball team's team fit and personal resilience, which is of great significance to the training of volleyball players.

To study the improving the performance of cooperative spectrum sensing, Yao et al. consider a cluster-based cooperative spectrum sensing (CSS) scheme in the Energy Harvesting Cognitive Wireless Communication Network (EH-CWCN). Among them, the cognitive node (CN) clusters according to its received power level to improve the perception performance [1]. Its main research is the application of wireless sensor networks in cooperative spectrum sensing, but the tactical analysis model is not comprehensive enough. To improve the performance of the sports team, it is essential to analyze the team's tactics from the game video. Athlete's trajectory is the most useful tactical analysis clue in sports videos. Chen et al. proposed a technique to reconstruct player trajectories from broadcast basketball videos [2]. He proposed to obtain tactical information from the video, but the application of the wireless communication network is not complete. To study the application of wireless communication networks, Uddin proposed a two-hop wireless communication architecture for the smart grid (SG) composed of smart meters (SM), aggregators (AG), and cellular base stations (BS) [3]. The wireless communication architecture studied can be applied to the analysis of volleyball tactics studied in this article. The advancement of smart grids and the advocacy of “green communications” have inspired wireless communication networks to obtain energy from the surrounding environment and operate in an energy-saving manner to achieve economic and ecological benefits. Hu et al. conducted a contemporary review of the latest breakthroughs in the utilization, redistribution, trading, and planning of energy collected in wireless networks that interoperate with smart grids in the future [4]. It applies the wireless network to the smart grid, but it does not involve enough tactical analysis. Jokgu is a South Korean online sport that has both volleyball and football skills in the form of challenge skills and games. Chang et al.'s main research is that Jokgu provides students with opportunities to develop physical fitness components related to health and skills, such as eye-foot coordination, flexibility, kicking, and juggling basic motor skills [5]. It mainly describes a sport similar to volleyball. If it can increase the application of volleyball tactics, it will be more in line with the purpose of this article. To study motion capture technology, Fang et al. proposed a new type of data glove, which can capture the movement of the arms and hands through inertial and magnetic sensors [6]. The motion capture technology he studied can be used in the analysis of volleyball tactics, but the application of wireless communication networks is not complete. Optical motion capture is based on estimating the three-dimensional position of the marker through triangulation from multiple cameras. Rahimian and Kearney introduced and compared two camera placement methods. The first method is based on a metric that calculates the visibility of the target point in the presence of dynamic occlusion from a camera with a “good” view. The second method is based on the view distribution of the target point [7]. Although the motion capture method he designed can capture the motion of volleyball, it is not sufficiently applied in wireless communication networks. To study the application of wireless communication networks, Bhatnagar's work mainly focuses on the design and analysis of wireless communication networks. He also explored the spectrum and energy efficiency aspects of next-generation networks such as smart grid communications [8]. Its research on wireless communication networks is very in-depth, but it would be better if it can be applied in the analysis of volleyball tactics. All above documents are mostly about wireless communication networks and motion capture, which are relatively small in the analysis of volleyball tactics. This requires an in-depth understanding of the connotations of volleyball tactics and how to combine wireless communication networks to analyze volleyball tactics.

The innovation of this paper is to use the characteristics of network management and network objects in the wireless communication network to design a tactical analysis model based on the wireless communication network based on the LTE system and MIMO technology. Then, write volleyball tactics and game analysis into the tactical analysis model, and get the wireless communication network volleyball tactics analysis model studied in this paper. The innovation in the experiment of this paper is to design the scenario assignment problem simulation experiment, the algorithm simulation experiment, and the comparative investigation and analysis of the volleyball game, spiking technical ability, and optimize the volleyball tactics analysis model through the data obtained from the experimental analysis.

## 2. Method of Volleyball Tactics Analysis Model Based on Wireless Communication Network

### 2.1. Wireless Communication Network

The application of wireless communication network [9] is shown in Figure 1.

#### 2.1.1. Cognitive Radio

Cognitive radio (CR) [10] technology in a narrow sense refers to the detection of the user status of authorized spectrum resources by unlicensed users, without affecting the normal data communication of authorized users, opportunistic/shared/leased reuse of authorized spectrum for own data communication. Cognitive radio technology in a broad sense generally refers to nodes or subsystems in the network through sensing external environmental information, adaptively adjusting their own internal data transmission parameters (e.g., frequency band, transmit power, and beam direction) to improve the overall resource utilization efficiency of the network. The structure of the cognitive radio network is shown in Figure 2.

The classic cognitive wireless network model consists of two parts: a primary network and a secondary network. The primary network includes a primary user transmitter (PT) [11] and multiple primary user receivers (PR) [12]. For communication on the allocated authorized frequency band, the secondary network includes a secondary user transmitter (ST) and multiple secondary user receivers (SR). By detecting the use of the authorized spectrum, opportunistic/sharing/lease access to the authorized spectrum for own data communication. It can be seen from the description here that the research on cognitive wireless networks can be divided into two categories; one is the spectrum detection technology, and the other is the spectrum multiplexing technology.

*(1) Spectrum Detection*. The spectrum detection technology in the cognitive wireless network [9] is a signal detection technology born out of its own. Its goal is to determine the user status of the licensed frequency band by sampling and analyzing the transmission signal on the licensed frequency band. According to the different detection target nodes, cognitive network spectrum detection can be divided into main network sending node detection and main network receiving node detection. Since the receiving node does not send data, the commonly used receiving node detection method is to detect whether there is a corresponding receiving node in the coverage of the sending node by detecting the leakage of the local crystal oscillator (L0) at the radio frequency (RF) front end of the receiving node.

*(2) Spectrum Reuse*. Spectrum multiplexing technology refers to the cognitive network obtaining the access rights of the authorized spectrum through a certain method and carrying out its own data transmission under the premise of not affecting the normal communication of the main network. At present, spectrum multiplexing technology [13] can be roughly divided into spectrum sharing technology and spectrum collaboration technology. The former refers to the sharing of authorized spectrum resources by primary and secondary networks from the perspective of time division, frequency division, power division, or space division. The latter refers to the secondary network assisting the primary network in data transmission to obtain part of the spectrum resource utilization rights.

#### 2.1.2. Network Management and Network Objects

Network management [14] is to monitor and control the network. Network planning, network configuration, and network monitoring are the main functions of network management. Network planning refers to the planning the parameters required for the normal operation of the communication network according to the communication requirements. The network configuration is to set the planning parameters for the communication network equipment by realizing the parameter configuration means of the communication network connection. Network monitoring is the process of collecting network status information and providing corresponding feedback during network operations. The main functions of network management are shown in Figure 3.

#### 2.1.3. Overall Protection Framework

The LTE [15] access system must not only meet the security requirements of wireless network data transmission such as confidentiality, integrity, and antiforgery but also meet the security requirements related to wireless services. The LTE network needs to separately design the production control area and the management information area according to the characteristics of the different security zones of the network, focusing on protection in three parts: the main station side, the terminal side, and the boundary. The secure access scheme is mainly to provide a relatively secure communication channel between the system and the terminal and provide a safe and effective communication environment for network terminal users by using technical means such as identity authentication, data signature, and data encryption/decryption. Regardless of whether using an LTE public network or a private network, it should keep the gateway securely connected to the business network. LTE terminals should have information processing and calculation functions, two-way authentication, and encryption functions with low computational complexity.

The overall security protection architecture is divided horizontally into four parts: business layer, security access layer, LTE access layer, and terminal business layer in accordance with the principles of division, classification, and domain division. Vertically, it is divided into two major parts: production control area (I and II areas) and management information area (III, IV). Through this architecture system, it provides the required security protection requirements for LTE wireless networks. In the overall security protection architecture of the LTE wireless communication system, the service terminal layer at the bottom is composed of collection and detection terminals such as processing terminals, handheld mobile inspection terminals, sensor networks, and service terminals and is the source of service information data. The LTE access layer consists of four parts: a core network, a dedicated backhaul network, a base station, and a communication terminal, generally composed of software and hardware devices such as firewalls. The business layer is the data information control and processing center of the business layer and the main station platform of the business system.

To protect the user's true identity from being cracked during the LTE wireless transmission process, it then causes personal interest issues related to personal privacy and key information, each time the LTE network accesses the network, each user will be assigned a temporary identity GUTI corresponding to their real identity, which protects the real identity of the user in this way. Moreover, every time a user accesses the network, the network will assign an S-TMSI to the user as the identity of the user in this session. After the user accesses the network, the MME will generate a random number S-TMSI according to a preappointed random generation algorithm. The MME corresponds the generated random number S-TMSI with the real identity ID of the corresponding user. After the user access is completed, to protect the identity information from being leaked, the user uses the temporary identity assigned by the system for this session to perform data transmission with the mobility management entity. To ensure that both the user and the LTE network enjoy secure data transmission, identity authentication is required before the formal data transmission between the two, and the session key for this communication is negotiated during the authentication process.

#### 2.1.4. MIMO Technology

At present, the method of improving the system capacity can be summarized as follows: first is setting up more base stations, but the increase of base stations means the increase of communication cost, and the gain is not worth the loss. The second is to broaden the frequency band, but the available wireless frequency band resources are relatively limited; the third is to improve the spectrum efficiency, which has more practical significance than the previous two schemes in terms of cost and implementation. The structure of MIMO technology [16] is shown in Figure 4.

There are generally two ways to improve spectrum utilization efficiency. One is to increase the signal-to-noise ratio. According to the channel capacity formula, the signal-to-noise ratio is increased by 3 dB, and the channel capacity can be increased by 1 bit/s/Hz. Increasing the signal-to-noise ratio needs to increase the amplification power, but the existing power amplifiers are difficult to meet the requirements because it is difficult for the amplifier to maintain high power transmission in a wide linear range. At the same time, the heat dissipation of the device needs to be considered when the power is high.

In the traditional wireless communication system, there will be multipath propagation due to the characteristics of the wireless channel during the transmission process, and the multipath propagation will cause the energy of the wireless signal to fade rapidly, which will seriously affect the transmission performance of the system. The MIMO technology uses multiple antennas at both the transmitting end and the receiving end, which can effectively utilize multipath propagation, eliminate the impact of multipath propagation on system performance, and improve system performance. At the same time, MIMO technology can provide the system with spatial multiplexing gain to increase the capacity, eliminate the influence of wireless channel multipath and time-varying fading, enhance the reliability of signal transmission, and reduce the spatial diversity gain of transmission error rate.

MIMO technology can increase the system capacity, but the premise is that the subchannels need to be independent of each other, and at the same time, the physical adjacent antenna spacing between the transmitting end and the receiving end is required to be large enough, to prevent excessive correlation between received signals. However, it is difficult to install multiple antennas for mobile terminals and electronic devices that currently require small volumes.

### 2.2. Volleyball Tactics

#### 2.2.1. Tactical Analysis

Tactics [17], as an important part of the capability of sports competition itself, often appears in the field of military science, and it is also a professional term in this field. The objective reality of the existence of things is the basis of tactics. When a war occurs, the use of tactics is essential, and the tactics directly reflect the laws of war itself. Social productivity has progressed with the development of the times, and the material conditions determined by productivity are also gradually developing.

Based on the characteristics of volleyball games, this article believes that volleyball tactics are mainly reflected in the following aspects.

*(1) The Internal Laws of Different Manifestations in the Use of Volleyball Tactics*. With the continuous development and progress of society, volleyball is also constantly advancing, and the competition has become increasingly fierce. The level of all players has improved in varying degrees, which has intensified the intensity of the competition. If volleyball players want to achieve excellent sports performance, they must constantly master the tactical expressions such as the game play used in the volleyball game. According to the characteristics of one's own position, the key to master the tactical application form, in ordinary training, it is necessary to develop high-efficiency contact according to the position and focus.

The use of the above tactics requires athletes to fully master the inherent laws of these tactics, improve tactical awareness, accurately predict the opponent's intentions, and take corresponding actions in time to achieve ideal results.

*(2) Familiar with the Problems That Should Be Paid Attention to in Tactical Cooperation*. The expression of tactics is abstract and concise in the theory of written expression, but it is more complicated in actual application, and there are many changes in actual application. To use these tactics flexibly and accurately under these changing and complex circumstances, higher requirements are put forward for the application.

During the volleyball game, the situation on the game field changes rapidly. Due to the influence of many factors, the effects achieved by the tactics used by the athletes also change. Every sports team and athlete has its own tactical style of play, and there is a problem of mutual growth and mutual restraint. Based on the consideration of these issues, to achieve excellent sports performance in the game, defeat the opponent, and win the game, it is necessary to have a comprehensive and profound understanding and mastery of the tactical manifestations and characteristics of the team. At the same time, we must carefully study and understand the opponent's tactical play and performance characteristics and adopt threatening tactical cooperation to defeat the enemy, actively attack and defend, fight hard, gain the advantage of the game, and keep it.

*(3) Keen Observation and Prediction Ability*. The volleyball match is a contest between two sports teams. The victory of the match depends not only on one's own performance level but also on the overall performance of the opponent in the game. Tactics are used during the confrontation between the two teams. Without confrontation, there is no use of tactics. In the game, it is necessary to use tactical forms and tactical cooperation consciously and rationally. According to the performance of the opponent, choose one's own tactics in a targeted manner and defeat the enemy; only in this way, we can win the game. During the fierce competition, the competition was carried out with high intensity and tension, and the changes were very rapid. During the game, it is necessary to observe and predict the opponent's situation in a timely and accurate manner, accurately judge the opponent's intentions, adjust their own response measures in time, and take targeted measures to resist the opponent's attack. There will be many unexpected accidents during the game. We must have sharp observation and prediction ability for these emergencies to be able to deal with them in time and make correct and timely action measures. Therefore, keen observation and prediction ability play an important role in the application of volleyball game tactics.

#### 2.2.2. Game Theory

Game theory [18] particularly emphasizes that the possible reactions of competitors must be considered when formulating strategies, to adjust their actions according to the reactions of competitors and to maximize the interests of individuals or collectives. Its main application areas are shown in Figure 5.

*(1) The Basic Elements of the Game Model*. Game theory uses mathematical analysis to express its game model. The manifestations of game theory can be divided into standard and extended forms. Although game theory can be different in form, any game theory must have its basic elements, including as follows:

1. Players in the game. Players in the game refer to the participants who have the right to make their own decisions
2. Strategy set, which is also called strategy space
3. Payout function. The payout function in game theory can also be called the profit function or utility function of each player

*(2) Cooperative Game*. In a cooperative game [19], all game participants obey the game rules to make rational decisions, while the latter mainly studies the game participants to make game decisions without considering the impact on other participants. In the cooperative game, each participant is rational, emphasizing the overall fairness, and its Nash equilibrium is the state where the overall benefits are maximized.

In a static game, the players in the game make the game strategy at the same time or the two sides of the game make the game strategy without knowing what actions each other will take. In a dynamic game, all participants make game strategies one after the other, knowing the actions of both parties in the game. That is, in the dynamic game, the two sides of the game only act on the basis of information sharing.

The complete information game means that the players in the game can make the second round of game strategy only after they have fully grasped the game information. If the players do not have all the information of the game, or only understand part of the information, it will lead to some games with incomplete information, which is the game of incomplete information.

#### 2.2.3. Game Analysis of Volleyball Tactics

Individuals or collectives (such as institutions, companies, governments, and countries) who can independently choose strategies and implement them in game activities and can independently bear the corresponding game results are called game parties. In the “Prisoner's Dilemma,” although the police formulated the rules of the game, they themselves did not participate in the decision-making process and did not assume the corresponding game results. Therefore, the police cannot be regarded as a game player by definition. Two teams participating in a volleyball match can be regarded as two opposing players. Although the volleyball game is a collective confrontation event, once one party confirms to choose a certain tactic, it immediately needs the whole team to cooperate and complete the implementation of the tactic. That is, the selection and implementation of the strategy of the entire volleyball team are consistent. And regardless of whether the game wins or loses, the whole team jointly assumes the result of the game, which also satisfies the above description of the definition of the game party.

However, due to the dynamic nature of game activities, the process will interact and influence each other due to the different strategies chosen by different players. Therefore, the more parties participating in the game, the more difficult it is to analyze the game process, and the entire game process may therefore exhibit different attributes and characteristics. For this reason, when studying game problems, game activities are often divided into “single-player games,” “two-player games,” and “multiplayer games” according to the number of players participating in the game. The “person” here does not necessarily refer to a single individual person but the aforementioned game party.

Single-player game means that only one player participates in the game activity. Compared with two-player games and multiplayer games, the game process of single-player games is much simpler. Because the single-player game process in competitive volleyball is difficult to clarify, the volleyball player's choice of serve in daily training is used to establish a model to clarify the single-player game in volleyball.

The serving practice in the competitive training of volleyball players can be regarded as a single-player game played by the players themselves. For example, athletes have two options when serving the ball: one is to jump and serve vigorously, and the other is to jump and serve floating. The strong jump serve is strong and fast, which poses a greater threat to the opponent, but it also increases the risk of own mistakes accordingly. The miss rate of jump serve is low. Although the flight path of the ball is erratic, it poses relatively little threat to the opponent. It is suitable for targeted serve to find someone or find area tactics. During training, athletes will choose the way of serving practice according to their own technical characteristics, physical stamina, and combined with tactical needs. We assume that athletes who practice serving have two strategies to choose from: vigorously jump serve and jump serve float. A straight jump serve or a straight jump serve can make one satisfied, while the diagonal line fails to achieve the training goal, which is not satisfied, and it cannot get a sense of self-identity.

### 2.3. System Model and Outage Probability

The system model of a full-duplex single-carrier single-antenna SG relay is shown in Figure 6. The entire relay system is composed of source node *L*, relay node *E*, and destination node *S*. The transmitter (or receiver) of each node has only one antenna. Among them, the relay node *E* works in full-duplex mode, and while receiving the signal *a*_*L*_ transmitted by the source node, it also uses the same frequency to transmit the signal *a*_*E*_ to the destination node. Due to the imperfect self-interference cancellation technology, the relay node will also receive residual self-interference. In addition, assuming that the direct link from the source node to the destination node is weak but not negligible, the signal model of the entire relay system is

(1) $$\begin{array}{c} b=Ga+k. \end{array}$$

Among them, *b* = [*b*_*E*_, *b*_*S*_]^*T*^ represents the received signal, *a* = [*a*_*L*_, *a*_*E*_]^*T*^ represents the transmitted signal, *k* = [*k*_*E*_, *k*_*S*_]^*T*^ is additive white Gaussian noise, and *G* is the channel matrix. The relay system shown in Figure 6 is a double-hop system; that is, it contains only one relay node, so the channel matrix *G* can be equivalent to the following 2 × 2 dimensional form

(2) $$\begin{array}{c} G=\left[\begin{array}{cc} f_{LE} & f_{EE}\\ f_{LS} & f_{ES} \end{array}\right]. \end{array}$$

Assuming all channels

(3) $$\begin{array}{c} f_{xy}\left(x\in \left\{L,E\right\},y\left\{E,S\right\}\right). \end{array}$$

They are all Rayleigh fading channels; that is, the channel parameter *f*_*x*,*y*_ obeys the cyclic symmetric complex Gaussian distribution, and the amplitude∣*f*_*xy*_∣of the channel parameter obeys the Rayleigh distribution, and its probability density function (PDF) is

(4) $$\begin{array}{c} f_{\left|g\right|}\left(a\right)=\frac{2a}{\Omega_{xy}}q^{-a^{2}/\Omega_{xy}}. \end{array}$$

Among them, *Ω*_*xy*_ is the mean square error of ∣*f*_*xy*_∣.

Let *s*_*i*_ represent the transmit power of node *E*_*i*_, namely

(5) $$\begin{array}{c} \varepsilon \left\{{\left|a_{E_{i}}\right|}^{2}\right\}=q_{i}. \end{array}$$

Then, the SNR and the average SNR of the signal received by the node *E*_*i*_ transmitting node *E*_*j*_ are, respectively

(6) $$\begin{array}{c} \gamma_{xy}=\frac{{\left|f_{xy}\right|}^{2}q_{i}}{\sigma^{2}},\\ \bar{\gamma_{xy}}=\frac{\Omega ,yq_{i}}{\sigma^{2}}. \end{array}$$

Among them, *σ*^2^ is the power (variance) of the additive white Gaussian noise, *γ*_*xy*_ obeys the exponential distribution, and its probability density function is

(7) $$\begin{array}{c} f_{\gamma }\left(\gamma_{xy}\right)=\frac{1}{\bar{\gamma_{xy}}}e^{-\gamma_{xy}/\bar{\gamma_{xy}}}. \end{array}$$

Its cumulative distribution function (CDF) is

(8) $$\begin{array}{c} F_{\gamma }\left(\theta_{xy}\right)=\int_{0}^{\theta_{xy}}f_{\gamma }\left(\gamma_{xy}\right)d\gamma_{xy}=1-e^{-\theta_{xy}/\bar{\gamma_{xy}}}. \end{array}$$

In the relay system, the relay node *E* can receive the desired signal from the source node and the residual self-interference signal at the same time, and the destination node *S* can receive the desired signal from the relay node and the direct signal from the source node at the same time. Assuming that the signal from the source node to the destination node is weak, but not negligible, and the relay system does not adopt the joint coding scheme of the source node and the relay node, the SINR of the signal received by the relay node *E* and the destination node *S*, respectively

(9) $$\begin{array}{c} \gamma_{E}=\frac{{\left|f_{LE}\right|}^{2}qL}{\sigma^{2}+{\left|f_{EE}\right|}^{2}qE}=\frac{\gamma_{LE}}{1+\gamma_{EE}},\\ \gamma_{S}=\frac{{\left|f_{ES}\right|}^{2}qE}{\sigma^{2}+{\left|f_{LS}\right|}^{2}qL}=\frac{\gamma_{ES}}{1+\gamma_{LS}}. \end{array}$$

At this time, the end-to-end channel capacity of the SG relay system is

(10) $$\begin{array}{c} Z=\min\left\{Z_{LE},Z_{ES}\right\}=\min\left\{\log_{2}\left(1+\gamma_{E}\right),\log_{2}\left(1+\gamma_{S}\right)\right\}. \end{array}$$

If the end-to-end capacity of the system cannot reach the given target information rate *E*, an outage occurs. The outage probability of the SG relay system is

(11) $$\begin{array}{c} Q_{0}=U\left\{Z<E\right\}. \end{array}$$

It is equivalent to the interruption of the source node to the relay node (the *L*-*E* link is interrupted) or the relay node to the destination node (the *E*-*S* link is interrupted), that is,

(12) $$\begin{array}{c} Q_{0}=1-\left(\left.1-U\left\{Z_{LE}<E\right\}\right)\left(1-U\right.\left\{Z_{ES}<E\right\}\right), \end{array}$$

making

(13) $$\begin{array}{c} \gamma_{th}=2^{E}-1. \end{array}$$

Then, *γ*_*th*_^2^ is the SINR required to reach the target information rate, so the system interruption can be equivalent to the relay node's SINR*γ*_*E*_ not satisfying *γ*_*th*_ or the destination node's SINR*γ*_*S*_ not satisfying *γ*_*th*_, so there is

(14) $$\begin{array}{c} Q_{0}=1-\left(\left.1-U\left\{\gamma_{E}<\gamma_{th}\right\}\right)\left(1-U\right.\left\{\gamma_{S}<\gamma_{th}\right\}\right). \end{array}$$

Among

(15) $$\begin{array}{c} U\left\{\gamma_{E}<\gamma_{th}\right\}. \end{array}$$

That is, the probability that the link between the source node and the relay node is interrupted, and *U*{*γ*_*S*_ < *γ*_*th*_} is the probability that the link between the relay node and the destination node is interrupted.

For the probability *U*{*γ*_*E*_ < *γ*_*th*_} that the link from the source node to the relay node is interrupted is

(16) $$\begin{array}{c} U\left\{\gamma_{E}<\gamma_{th}\right\}=1-\frac{1}{1+\left(\gamma_{th}\bar{\gamma }EE/\bar{\gamma }L,E\right)}e^{-\gamma_{th}/\bar{\gamma }L,E}. \end{array}$$

In the same way, the probability *D*{*γ*_*S*_ < *γ*_*th*_} that the link between the relay node and the destination node is interrupted is

(17) $$\begin{array}{c} U\left\{\gamma_{S}<\gamma_{th}\right\}=1-\frac{1}{1+\left(\gamma_{th}\bar{\gamma }LS/\bar{\gamma }ES\right)}e^{-\gamma_{th}/\bar{\gamma }LES}. \end{array}$$

Incorporating formula (16) and formula (17) into formula (14), the end-to-end outage probability of the full-duplex SG relay system is finally obtained as

(18) $$\begin{array}{c} Q_{0}=1-\frac{1}{1+\left(\gamma_{th}\bar{\gamma }EE/\bar{\gamma }L,E\right)}e^{-\gamma_{th}/\bar{\gamma }L,E}1-\frac{1}{1+\left(\gamma_{th}\bar{\gamma }LS/\bar{\gamma }ES\right)}e^{-\gamma_{th}/\bar{\gamma }LES}. \end{array}$$

## 3. Volleyball Tactics Analysis Simulation Test Experiment Based on Wireless Communication Network

### 3.1. Simulation Experiment of Scene Allocation Problem

China mobile's wireless network planning index requirements are shown in Table 1.

China Unicom's wireless network planning index requirements are shown in Tables 2–4.

China telecom's LTEFDD wireless network planning index requirements are shown in Table 5.

Considering the comparison of the social utility and spectrum utilization performance of each algorithm in a simplified scenario, it is assumed that the central decision-maker divides the frequency range into 144 continuous subintervals. The maximum number of requirements for each secondary user frequency subinterval is 36, and each secondary user randomly selects the number of requirements on [1,36] and normalizes the quotations of secondary users to a uniform distribution on [0,1]. At the same time, because the WSDP-S problem is a special case of the WSDP problem, the latter can also be used to simplify performance comparisons in scenarios.  Figure 7 shows a comparison of social utility in a simplified scenario. Among them, the abscissa is the number of secondary users, the ordinate is the social utility, and the curve represents the relationship between the social utility of different algorithms and the number of secondary users.

Figure 7 shows a comparison of spectrum utilization in a simplified scenario. The spectrum utilization of each algorithm increases as *n* increases. Among them, the spectrum utilization rate under the optimal solution is not the highest, which can be considered as a trade-off between spectrum utilization rate and social utility.

### 3.2. Algorithm Simulation Experiment

This article simulates a communication system topology with 2 hotspots, and the *α* value of each base station is set to 0.5. That is, the zero-load power of each base station is half of its maximum operating power, and each base station has 2000 resource blocks to meet user needs. The simulated scene data is as follows: the area of the area is 2∗2 square kilometers, there are a total of 60 base stations in the area, the coverage radius of each base station is 200 to 400 meters, and the number of simulated users ranges from 1,000 to 20,000. The path loss model adopted is *l*(*dB*) = 35.2 + 35log_10_(*d*), where *d* represents the distance from the user to the base station in meters.

The users are uniformly distributed in the area, and the user's signal-to-noise ratio (SNR) can be derived based on the distance from the base station and the path loss model, as shown in Figure 8.

As can be seen from Figure 8, the power savings of these two algorithms decrease as the number of users increases. This is because as the number of users increases, the load of the base station increases, and more base stations must be in operation to ensure the quality of service for users. The algorithm proposed in this paper saves more power. This is because the distributed access algorithm calculates the utility value of the mobile device at the same time, so it may produce a ping-pong effect, which makes the mobile station switch infinitely between the original base station and the target base station. The algorithm proposed in this paper can effectively avoid this problem. On the other hand, each base station can determine by itself whether it should be shut down. It can be seen that more base stations can be shut down using the algorithm proposed in this paper, so the energy saving is higher.

## 4. Improved Results of Volleyball Tactics with Wireless Communication Networks

### 4.1. Comparative Investigation and Analysis of Volleyball Spiking Technical Ability

Smashing is the basic technique of volleyball, and it is also the most powerful technique among the various techniques of volleyball. It is the main means of scoring in the game. The ability level of the spiking technique, which can best show the offensive ability of a team, is the key to victory in the game. Therefore, this paper investigates and analyzes the data of four groups of college volleyball matches, and the results are shown in Figure 9.

From the spiking data in Figure 9, it can be seen that the total spiking success rate of the first group of universities is 59%, and the total spiking success rate of the second group of universities is 53.27%. The third group of universities has a spiking success rate of 42.07%, and the fourth group of universities has a total spiking success rate of 48%.

### 4.2. Test Analysis of Volleyball Tactics Analysis Model Based on Wireless Communication Network

This paper optimizes the volleyball tactics analysis model of the wireless communication network through the data collected in the experiment. To explore the effect of the optimized volleyball tactics analysis model on volleyball matches, this article compares 20 volleyball teams into two groups. One group is a control group, which only conducts ordinary training; the other group is an experimental group, which conducts volleyball tactics analysis and model training based on wireless communication network. Taking its team fit and on-the-spot adaptability as the evaluation criteria, the results of the experiment were recorded, and the results of the experiment are shown in Figure 10.

It can be seen from Figure 10 that the control group is traditional volleyball tactical training, and its team fit is only 71.02%, while the experimental group based on the wireless communication network-based volleyball tactical analysis model training has a team fit of 93.14%, an increase of 22.12%. The traditional volleyball tactics training individual on-the-spot adaptability is only 81.65%, while the experimental group based on the wireless communication network-based volleyball tactical analysis model training individual on-the-spot adaptability can reach 90.7%, an increase of 9.05%. This shows that the volleyball tactics analysis model based on the wireless communication network can very effectively improve the team fit of the volleyball team, and it can also improve the individual resilience of the team by a small amount.

## 5. Conclusions

This article mainly studies the establishment of the volleyball tactics analysis model based on the wireless communication network, so this article combines the characteristics of the radio network and the characteristics of the wireless communication network and accesses the LTE system. Based on the MIMO technology, the tactical analysis model of the wireless communication network is established, and then, the tactical analysis model of the wireless communication network is optimized for the tactics and games of volleyball training. Then, carry out simulation test experiments on the wireless communication network to further optimize the performance of the wireless communication network, and then, further optimize the volleyball tactical analysis model of the wireless communication network through the data of specific volleyball games. The final volleyball tactics analysis model can effectively improve the team fit of the volleyball team, and it can also improve individual on-the-spot adaptability.

## Figures and Tables

**Figure 1:** Application of wireless communication network.

**Figure 2:** Cognitive radio network structure.

**Figure 3:** Main functions of network management.

**Figure 4:** Structure of MIMO technology.

**Figure 5:** Application areas of game theory.

**Figure 6:** Full-duplex single-antenna single-carrier DF relay system model.

**Figure 7:** Comparison results of social utility and spectrum utilization in a simplified scenario: (a) comparison of social utility in simplified scenarios; (b) comparison of spectrum utilization in simplified scenarios.

**Figure 8:** Simulation experiment results: (a) the impact of the number of users on power consumption; (b) proportion of base stations closed.

**Figure 9:** Comparison results of spiking techniques in colleges and universities: (a) anticounterfeiting situation comparison; (b) comparison of the first attack situation.

**Figure 10:** Experimental comparison results: (a) team fit; (b) on-the-spot adaptability.

**Table 1:** China mobile TD-LTE wireless network planning index requirements.

Type	Penetration loss	RSRP		RS-SINR	Coverage	Cell edge rate
		*F* band	*D* band			
Main city	High	>-100	>-98	>-3	95%	1
Main city	Low	>-103	>-101	>-3	95%	1
General urban area		>-103	>-101	>-3	95%	1
County and suburbs		>-105	>-103	>-3	95%	1

**Table 2:** China Unicom LTEFDD wireless network planning index requirements.

Area type	RSRP	RS-SINR	Coverage	Cell edge rate	Average cell throughput
Dense urban area	>-100	>-5	90%	DL/UL:4/1	DL/UL:35/25
General urban area	>-100	>-5	90%	DL/UL:4/1	DL/UL:35/25
Tourist attraction	>-105	>-5	90%	DL/UL:4/1	DL/UL:30/20
Airport express, high-speed rail	>-110	>-5	90%	DL/UL:2/0.512	DL/UL:25/15

**Table 3:** China Unicom TD-LTE wireless network planning index requirements.

Area type	RSRP	RS-SINR	Coverage	Cell edge rate	Average cell throughput
Dense urban area	>-105	>-5	90%	DL/UL:1/0.128	DL/UL:18/10
General urban area	>-105	>-5	90%	DL/UL: 1/0.128	DL/UL: 18/10
Tourist attraction	>-110	>-5	90%	DL/UL: 1/0.128	DL/UL: 18/10

**Table 4:** China Unicom U900 wireless network planning index requirements.

Area type	RSCP	Ec/Io	Coverage
County town	>-90	>-12	90%
Suburban township	>-95	>-14	90%
Rural area	>-100	>-14	90%
Airport express, high-speed rail	>-90	>-12	90%
Provincial high-speed, high-speed train	>-95	>-12	90%
Other roads	>-95	>-14	90%

**Table 5:** China telecom LTEFDD wireless network planning index requirements.

Area type	RSRP	RS-SINR	Coverage	Cell edge rate
Dense urban area	>-105	>-3	97%	DL/UL:4/0.256
General urban area	>-105	>-3	96%	DL/UL:4/0.256
Suburbs, county towns	>-105	>-3	95%	DL/UL:4/0.256

## Data Availability

All the data used is given in the paper.
